# Effect of WeChat-Based Health Preaching Combined with an Enhanced Recovery after Surgery Model on Perioperative Limb Motor Function and Complications in Orthopaedic Patients

**DOI:** 10.1155/2022/9538138

**Published:** 2022-03-08

**Authors:** Zhijuan Pang, Bin Hu, Dejun Chai, Ping Li, Le Ma, Lei Liu, Wei Li

**Affiliations:** ^1^Department of Rehabilitation, The 2nd Affiliated Hospital of Qiqihar Medical University, Qiqihar 161000, Heilongjiang Province, China; ^2^Department of Neurology, The 2nd Affiliated Hospital of Qiqihar Medical University, Qiqihar 161000, Heilongjiang Province, China

## Abstract

**Objective:**

To evaluate the effect of WeChat-based health preaching combined with an enhanced recovery after surgery (ERAS) model on perioperative limb motor function and complications in orthopaedic patients.

**Methods:**

By means of retrospective analysis, the medical data of 68 orthopaedic patients who received surgical treatment in our hospital (from 01, 2020–12, 2021) were collected, and the patients were equally divided into the study group (SG) and control group (CG) according to their admission order, with 34 cases each. From 7 d before surgery to the time of hospital discharge, WeChat-based health preaching combined with ERAS perioperative nursing was performed to patients in the SG, and routine orthopaedic perioperative nursing was performed to those in the CG. Before and after nursing, patients' Visual Analog Scale for Fatigue (VAS-F) scores, Houston Pain Outcome Instrument (HPOI) scores, and brief Fu-gI-Meyer (FMA) motor scores were investigated and the incidence rates of postoperative complications and nursing satisfaction of patients in the two groups were recorded.

**Results:**

After nursing, SG obtained a significantly better VAS-F score and HPOI score (*P* < 0.001), significantly higher postoperative 7 d and predischarge lower limb FMA scores (20.06 ± 2.13 vs 18.38 ± 2.36, 27.50 ± 1.90 vs 24.09 ± 2.25, *P* < 0.05), and significantly lower annual incidence rate of complications compared with those of the CG (*P* < 0.05); and the nursing satisfaction scores of the SG and CG were 9.18 ± 0.82 points and 6.76 ± 0.91 points, respectively, indicating significantly higher nursing satisfaction in the SG than in the CG (*P* < 0.001).

**Conclusion:**

The nursing model of WeChat-based health preaching combined with ERAS can effectively improve the knowledge level of orthopaedic patients, thereby improving their abilities of pain management and self-management, accelerating the recovery of their limb function, and reducing the incidence rate of postoperative complications. The patients are more satisfied with such nursing model, indicating its better promotion value.

## 1. Introduction

Orthopaedic rehabilitation is the discipline that specifically provides comprehensive rehabilitation intervention for patients with orthopaedic injuries, aiming to help the patients' affected limb recover and restore their normal life ability through surgery, functional exercise, etc. [1] As the medical concept continues to advance in recent years, the enhanced recovery after surgery (ERAS) model has been gradually applied in orthopaedic rehabilitation, which is based on evidence-based medicine, in which medical staff from multiple disciplines are jointly involved to formulate a perioperative intervention plan with a view to reduce the physiological and psychological traumatic stress reaction of patients through pain control, nutritional support, venous thrombo prophylaxis, and other measures [2, 3], thus improving their postoperative pain sensation and reducing the complication rate. Although most studies have shown a significant value of the ERAS model in the early postoperative rehabilitation of orthopaedic patients [4], Laura et al. suggested that there are multiple limitations to the application of this model in practice and more than 37.6% of patients cannot really benefit from it [5]. Meta-analysis confirmed that the limiting factors of the ERAS model include the subjective motility of patients in addition to multidisciplinary conceptual differences, and subjective motility is a key element influencing the efficacy of perioperative nursing implementation under the ERAS model [6] because poor subjective motility leads to declined enthusiasm in compliance with perioperative nursing measures under the ERAS model and then causes failure to exert corresponding effects of the model. Scholars Sattler et al. reported that rehabilitation self-efficacy of patients with early ambulation after a hip replacement was significantly higher than that of patients without early ambulation, indicating that good rehabilitation self-efficacy is the key to improving patients' subjective mobility [7]. Self-efficacy is a direct manifestation of patients' confidence in rehabilitation and is closely related to patients' level of health knowledge [8]. Patients with low levels of health knowledge often fail to clearly recognize the positive effect of the ERAS model, and most patients tend to believe that bed rest should be taken after an injury because rest is more conducive to limb recovery, so they have poor subjective motility and nursing compliance and are unwilling to effectively go along with the nursing measures under the ERAS model [9, 10]. Providing patients with scientific and efficient health education can improve their health knowledge levels and enhance their rehabilitation self-efficacy, thus improving the outcomes of perioperative nursing under the ERAS model. Conventional oral preaching is easily affected by the communication ability of nursing personnel, it is difficult for nursing personnel to grasp the correct timing of preaching, and the content of which is often contrary to the actual needs of patients, so the preaching effect is unsatisfactory. WeChat has now become an important tool in the daily communication of Chinese residents, and a large number of studies have shown that WeChat-based health preaching can effectively improve patients' health knowledge levels. However, at the current stage, there has been no study to apply it in the perioperative nursing of patients under the ERAS model. Based on this, the effects of WeChat-based health preaching combined with the ERAS model on orthopaedic patients was explored herein, with the results summarized as follows.

## 2. Materials and Methods

### 2.1. General Data

By means of a retrospective study, the medical data of 68 orthopaedic patients who received surgical treatment in our hospital (from 01, 2020 to 12, 2021) were analyzed, and the patients were equally divided into the study group (SG) and control group (CG) according to their admission order, with 34 cases each. Compared between the SG and CG, no statistical differences in patients' general data were observed (*P* > 0.05), including gender (19 males and 15 females vs 20 males and 14 females), age (39.74 ± 7.40 vs 39.24 ± 8.25 years), body mass (62.46 ± 3.38 vs 62.27 ± 3.16 kg), course of disease (3.68 ± 1.30 vs 3.62 ± 1.09 d), number of cases with upper limb fractures (17 vs 18), and number of lower limb fractures (17 vs 16).

Inclusion criteria: (1) the patients were diagnosed with traumatic fracture [11]; (2) the patients' comprehensive ability, language expression ability, and writing ability met the study requirements; (3) the patients were over 18 years old; (4) the patients had complete clinical data; (5) the patients did not have vascular occlusive diseases for nearly half a year; and (6) the patients did not have coagulation disorders. Exclusion criteria: (1) the patients had limb motor dysfunction before fracture; (2) the patients had severe osteoporosis; (3) the patients had off-bed activity contraindication; (4) the patients had chronic pain in the past; (5) the patients had mental diseases, etc. and could not communicate with others; (6) the patients had undergone orthopaedic surgery in nearly half a year; and (7) the patients were complicated with other organic diseases that might affect the study results.

### 2.2. Study Design

The study met the principles in *World Medical Association Declaration of Helsinki (2013)* [12], and its nature was a retrospective study. After enrollment, the patients understood the study objective and signed the informed consent.

### 2.3. Methods

Routine orthopaedic perioperative nursing was conducted to patients in the CG. Various examinations were conducted and patients were guided to undergo fasting and water deprivation before surgery, and the data of their vital signs were closely monitored during surgery. Because of the thin hospital gown for patients undergoing orthopaedic surgery and skin exposure, most patients had lower skin temperature and were easy to have venous stasis and decreased blood oxygenation capacity of local tissues, so the nursing personnel should pay attention to patients' body temperature changes and ensure that the operating room temperature and humidity were within the appropriate range. After surgery, the nursing personnel repeatedly advised the patients to keep warm, adjusted the ward temperature, and encouraged the patients to do early off-bed activity.

For patients in the SG, WeChat-based health preaching combined with ERAS perioperative nursing was carried out, namely, the following measures were taken on the basis of the CG: (1) Establishment of a WeChat group: staff from rehabilitation, neurology department, and other disciplines were included in the team and were invited to the WeChat group on the day that patients agreed to join the study, and patients should grasp the basic use of the WeChat group and official account, if not, education was conducted; WeChat was always adopted to maintain a good and effective communication with the patients except face-to-face communication at all stages from admission to discharge. (2) Preoperative nursing: ① before surgery, patients were informed of the ERAS concep, and familiarized with the surgery plan and rehabilitation plan to alleviate their fear and enhance their confidence in the treatment; ② knowledge related to orthopaedic surgery was pushed to patients via articles of the official account, precautions of perioperative period were informed of the patients in the WeChat group every night, and such articles and messages should be sent when the patients were not at rest; ③ patients were graded according to their condition, primary evaluation and preaching was performed to high-risk patients, and in the form of video education, patients were guided online to actively treat their principle illness, so that they could understand the negative impact of principle illness, complications, and adverse mental status on rehabilitation before surgery; ④ before surgery, pain control education was performed to explain the method for alleviating pain, a multimode analgesic method was adopted in the perioperative period, and postoperative analgesic nursing was conducted to patients according to their pain sensation, and at the same time, patients received a music therapy, relaxation therapy, and other therapies to ease pain; ⑤ patients could eat nonsolid food 6 h before surgery and drink 10% dextrose solution 4 h before surgery; current studies showed that postoperative early water and food consumption could reduce the incidence rate of hypopotassemia, accelerate gastrointestinal tract recovery, and therefore the nursing personnel needed to prepare a targeted healthy recipe according to patients' food preference, and provide early nutrition support for patients; ⑥ the questions raised by patients in the WeChat group were answered in time to reduce their doubts. (3) Postoperative nursing: ① complication prevention was re-emphasized through pushing articles of the official account to inform patients about ways to prevent various types of complications and improve their self-management ability and crisis awareness; ② after surgery, patients who underwent orthopaedic surgery required bed rest, and reduced activity caused a slower venous return rate and then led to complications such as venous thrombosis, so after easing pain, patients should be encouraged to do off-bed activities and proper functional exercises to improve blood circulation; the nursing personnel should make rehabilitation exercise videos and send it to patients via the official account and WeChat group, so as to remind the patients of the necessity of early off-bed activities; e.g., early postoperative muscle contraction exercise and regular turning over could effectively promote venous return, and the patients were encouraged to finish daily attendance of exercise and communicate their status of doing functional exercises in the WeChat group; ③ all nursing personnel passed the pain knowledge training, and informed the patients of the usage of an analgesic pump and the possible analgesic-induced adverse reactions in the form of video education to improve patients' pain management ability; if it was inconvenient for the patients in the SG to watch the educational video with their mobile phone, their family members could play it for them.

### 2.4. Observation Criteria

1. Visual Analog Scale for Fatigue (VAS-F) score [13]: the scale was used to evaluate patients' degree of fatigue before and after nursing, which is closely related to the patients' postoperative recovery status. VAS-F contained 18 items related to subjective experience of fatigue, and each item was corresponding to a visual analog line on a scale of 0–10 points for the patients to reflect their current feeling by drawing circles on it. In VAS-F, 0–2 points indicated no fatigue at all and 8–10 hours of sleep needed; 3–4 points indicated occasional fatigue and 11–14 hours of sleep needed; 5–6 points indicated feeling fatigue and 15–16 hours of sleep needed; 7–8 points indicated feeling weak and 17–18 hours of sleep needed; and 9–10 points indicated laziness to speak and more than 18 hours of sleep needed.
2. Houston Pain Outcome Instrument (HPOI) score [14]: the scale for pain control education satisfaction was selected in this study to evaluate patients' pain postoperative 7 d and before discharge and patients' satisfaction with pain control, which is conducive to the evaluation of the actual effect of WeChat-based health education. On a scale of 0–10 points, 0 point indicated pain not being alleviated and dissatisfaction with pain control education, and 10 points indicated pain being completely alleviated and total satisfaction with pain control education, with higher scores indicating higher satisfaction with pain control education.
3. Fu-gI-Meyer (FMA) score [15]: the scale was used to assess patients' upper and lower limb motor function postoperative 7 d and before discharge, with higher scores indicating lighter motor dysfunction. ① Upper limb motor function: assessment in sitting position, including reflex activity, flexor synergy, extensor synergy, activities accompanied by common movement, separation movement, normal reflex activity, wrist stability, joint flexion-extension of finger, and coordination and quick finger-nose test, with a total score of 66 points; ② lower limb motor function: assessment in spine position (reflex activity and flexor synergy, and coordination/speed test), sitting position (combined common movement and normal reflex) and standing position (separation movement), with a total score of 34 points.
4. Incidence rate of complications: after surgery, the numbers of occurring stage II and above joint stiffness, deep venous thrombosis, and pressure sore in patients were recorded monthly, and the annual incidence rates were recorded.
5. Nursing satisfaction: a scale for investigating nursing satisfaction was proposed by our hospital on a scale of 0–10 points, with higher scores indicating higher patient satisfaction with nursing.

### 2.5. Statistical Processing

In this study, the data processing software was SPSS20.0, the picture drawing software was GraphPad Prism 7 (GraphPad Software, San Diego, USA), the items included were enumeration data and measurement data, the methods used were *X*^2^ test and *t*-test, and differences were considered statistically significant at *P* < 0.05.

## 3. Results

### 3.1. Comparison of Patients' VAS-F Scores and HPOI Scores

After nursing, the VAS-F score and HPOI score were significantly better in the SG than in the CG (*P* < 0.001), see Figure 1.

### 3.2. Comparison of Patients' FMA Scores

After nursing, the FMA scores were significantly higher in the SG than in the CG (*P* < 0.05), see Figure 2.

Postoperative 7 d and before discharge, the upper limb FMA scores were significantly higher in the SG than in the CG (45.74 ± 2.29 vs 38.62 ± 2.25, 56.68 ± 2.25 vs 46.94 ± 2.30, *P* < 0.001); and postoperative 7 d and before discharge, the lower limb FMA scores were significantly higher in the SG than in the CG (20.06 ± 2.13 vs 18.38 ± 2.36, 27.50 ± 1.90 vs 24.09 ± 2.25, *P* < 0.05).

### 3.3. Comparison of Patients' Incidence Rates of Postoperative Complications

In the SG, there were 0 cases with stage II and above joint stiffness (0.0%), 1 case with deep venous thrombosis (2.9%) and 1 case with pressure sore (2.9%); in the CG, there was 1 case with stage II and above joint stiffness (2.9%), 3 cases with deep venous thrombosis (8.8%), and 4 cases with pressure sore (11.8%). The annual incidence rate of complications was significantly lower in the SG than in the CG (*P* < 0.05).

### 3.4. Comparison of Patient Satisfaction with Nursing

The nursing satisfaction score was significantly higher in the SG (9.18 ± 0.82 points) than in the CG (6.76 ± 0.91 points) (*P* < 0.001).

## 4. Discussion

Enhanced recovery after surgery (ERAS) is an emerging concept in the process of humanism development, which aims to reduce the stress reaction of patients and the incidence of postoperative complications, and accelerate the recovery process through health preaching, pain management, nutritional support, etc. [16]. Because the ERAS model is based on evidence-based medicine and has an ideal scientific nature and validity, it has now been widely used in the clinical nursing of gastric cancer, colorectal cancer, primary liver cancer, and other diseases [17]. Orthopaedic rehabilitation is an important part of the treatment of orthopaedic patients, the application of the advanced ERAS model is of great significance for their postoperative rehabilitation, and there have been a large number of studies combining the ERAS model with orthopaedic rehabilitation [18, 19]. However, Yu Guozhu et al. found that orthopaedic patients had low adherence to the ERAS model [20], and the vast majority of patients believed that staying in bed after surgery was more beneficial for the affected limb while avoiding the potential for secondary damage. It has been shown that prolonged bed rest can lead to joint stiffness and difficulty in mobility, and the patients' limb function is difficult to be improved in the optimal rehabilitation period. A report in the *Surgical Literature* has shown that patients' higher compliance with ERAS is associated with a more pronounced clinical benefit, and that a 50.0%–90.0% increase in the compliance rate can reduce the patients' perioperative complication rate by 20.0% and the length of hospital stay by 4 days [21], so improving patients' nursing compliance is key to improving the efficacy of perioperative nursing under the ERAS model.

Rehabilitation self-efficacy is a key element in determining nursing compliance. Self-efficacy refers to an individual's expected value for successful completion of an activity in a given context, which can directly or indirectly influence their behavioral performance, physiological function, and then affect the rehabilitation effect [22]. Patients' self-efficacy is influenced by various kinds of information, among which the most important influencing factor is cognitive level. Enhancing patients' health knowledge level through health preaching will not only be effective in elevating their expected values but also improve patients' nursing compliance in ways that enhance rehabilitation self-efficacy, making them more compliant with perioperative nursing under the ERAS model. The preaching model adopted for patients in CG in this study was conventional preaching, that is, oral preaching by the nursing personnel, which has the disadvantage of focusing on knowledge instillation, failing to establish an effective feedback mechanism, so patients can only listen to health knowledge unilaterally, and it is easy to cause situations in which the preaching content does not meet patients' actual needs. Not only that, the effect of oral preaching is limited by the knowledge level and language skills of patients and nursing personnel, so it is difficult for different patients to obtain the same preaching effect [23]. Compared with CG, the WeChat medium selected for SG is more real-time and effective. This software is an important way to improve the coverage of information, which can send orthopaedic rehabilitation information to patients according to different needs in the form of speech, video, text, etc. and is more conducive to understanding and acceptance of patients.

The study results showed that the VAS-F score and HPOI score were significantly better in the SG than in the CG after nursing (*P* < 0.001), indicating that the health knowledge education level was more desirable in the SG and that WeChat-based health preaching successfully avoided the disadvantages of obscure text and lacking patient feedback channel [24, 25], providing a good communication way for patients and nursing personnel. Close communication relied on WeChat can enhance patients' trust and satisfaction with the nursing personnel, alleviate patients' fear and doubt, which is conducive to maintaining a good nurse-patient relationship and elevating patients' compliance with perioperative nursing measures conducted by the nursing personnel. From the results of limb motor function recovery, it was concluded that the FMA scores were significantly higher in SG than in CG (*P* < 0.05), which was due to the fact that the promoted health knowledge level enabled enhancement of patients' postoperative self-management ability and pain control effects, so patients' subjective initiative in terms of rehabilitation intervention was increased obviously. On the basis of implementing the ERAS model during perioperative nursing, the enhanced self-management ability further reduced the incidence rate of complications, and therefore the annual incidence rate of complications was significantly lower in SG than in CG (*P* < 0.05).

In conclusion, the current ERAS nursing model has great potential, and enhancing the subjective motility of patients through health education is the key to the efficacy of the ERAS model, which is beneficial to meet the nursing needs of orthopaedic patients at present. WeChat-based health preaching combined with the ERAS model nursing can effectively improve the knowledge levels of orthopaedic patients, thereby improving their pain management and self-management abilities, accelerating the recovery of limb function, and reducing the incidence rate of postoperative complications. Patients are more satisfied with such a nursing model, indicating its good promotion value.

## Figures and Tables

**Figure 1:** Comparison of patients' VAS-F scores and HPOI scores (*x* ± *s*, points): (a) the VAS-F scores and (b) the HPOI scores. No significant differences in VAS-F scores and HPOI scores between the SG and CG before nursing were observed (2.97 ± 0.62 vs 3.00 ± 0.59, 2.12 ± 0.58 vs 2.12 ± 0.76, *P* > 0.05), and after nursing, the VAS-F score and HPOI score were significantly better in the SG than in the CG (1.26 ± 0.44 vs 2.09 ± 0.56, 6.88 ± 1.69 vs 5.03 ± 0.89, *P* < 0.001).

**Figure 2:** Comparison of patients' FMA scores (*x* ± *s*, points). (a) The upper limb FMA scores and (b) the lower limb FMA scores.

## Data Availability

The data used to support the findings of this study are available on reasonable request from the corresponding author.
